The article "Clinical Diagnosis of White Matter Softening in Premature Infants Based on Electroencephalogram (EEG)" was retracted in 2023. Reasons: signs of a paper mill; suspected computer-generated content; unreliable results or conclusions; concerns about the data.

# Clinical Diagnosis of White Matter Softening in Premature Infants Based on Electroencephalogram (EEG)

**DOI:** 10.1155/2021/6614191

**Published:** 2021-02-22

**Authors:** Li Hao, Lu Shen, Qigai Yin

**Affiliations:** ^1^Department of Neonatology, The First People's Hospital of Lianyungang, Lianyungang, Jiangsu 222002, China; ^2^Xuzhou Medical University Affiliated Hospital of Lianyungang, Lianyungang, Jiangsu 222002, China

## Abstract

Periventricular white matter softening in preterm infants can lead to severe sequelae and greatly affects the quality of life of preterm infants, and early diagnosis is of great clinical significance and value. The purpose of this study is to select a diagnostic test scientifically and rationally, to interpret and evaluate the results of the diagnostic test, and to evaluate the selected diagnostic method. Although DWI is a sensitive method for early diagnosis of PVL, it is not suitable for critical preterm infants. Therefore, according to clinical research data and the basic hardware conditions of our hospital, video EEG was chosen as the target diagnostic test method to explore whether VEEG can be used for early diagnosis of PVL. According to the results of this study, video EEG may play an important role in the early diagnosis of PVL, and it is believed that video EEG can be used as an auxiliary examination tool, especially for some critical preterm infants who are not suitable for DWI examination, and it can be used as an electrophysiological examination index for the preliminary diagnosis of periventricular white matter softening in preterm infants to indicate that the clinic should carry out necessary and appropriate diagnostic tests. The timely intervention and the results of VEEG are valuable for the assessment of the prognosis of critically ill preterm infants as raw data. However, the use of VEEG to screen clinically suspicious PVL preterm infants is a new attempt, and although good results have been achieved in foreign countries, this study has been conducted only recently in China and requires further exploration.

## 1. Introduction

Premature infants are at high risk for neurodevelopmental disorders of varying severity, and the most common brain injuries are periventricular-intraventricular hemorrhage (PIVH) and periventricular leukomalacia (PVL) [1]. PIVH is the main representative of hemorrhagic disorders of prematurity, and PVL is the characteristic form of ischemic brain injury in preterm infants. A large body of literature indicates that PVL is the most important neuropathological alteration of brain injury in preterm infants and is the most common form of brain injury in preterm infants weighing <1500 and <32 weeks of gestational age. PVL refers to the coagulative necrosis of the white matter with characteristic distribution, i.e., the dorsal white matter in the lateral horn of the lateral ventricle, especially involving the center of the semicircle, visual radiation, and auditory radiation [2]. It is the main cause of neurodevelopmental and behavioral disorders in surviving preterm infants and is an independent risk factor for cerebral palsy (cerebral palsy, CP), with the incidence of cerebral palsy reaching more than 60% in patients with typical PVL [3]. With the improvement in perinatal neonatal medicine, the success rate of rescue of critically premature infants has generally increased; however, the number of near and distant neurological abnormalities is still high, and the number of children disabled by PVL each year can reach more than 100,000, so the early diagnosis of periventricular white matter softening in preterm infants is worth exploring [4].

Periventricular white matter softening in preterm infants is usually asymptomatic and difficult to diagnose clinically; therefore, cranial imaging plays an important role in the early diagnosis of brain injury in preterm infants. The sensitivity and specificity of cranial CT for the early diagnosis of white matter lesions are low, and its diagnostic significance is not as high as that of ultrasound for early (edematous stage) and late (cystogenic stage) localized PVL. Brain ultrasound (US) is a practical diagnostic method in the neonatal period. It is simple, inexpensive, radiation-free, and has advantages for critically ill children who cannot be easily moved, and it is easy to follow-up regularly [5–10]. Brain ultrasound is sensitive and specific for the diagnosis of cystic PVL. However, diffuse PVL is more common than localized PVL, and when there are no cystic changes in the early stages of white matter injury, brain ultrasound is unspecific and can easily miss the diagnosis. Studies have shown that, in the early stage of PVL, brain ultrasound can only detect abnormal strong echoes in the lesion area with low sensitivity, and cannot diagnose PVL with diffuse PVL and softening lesions <0.5 cm. Previous studies have reported the limitations of brain ultrasound in the early diagnosis of PVL. Magnetic resonance imaging (MRI), as a noninvasive technique, has good density resolution of the gray and white matter of the brain, without the harm of X-ray radiation. In preterm infants, however, the water content in the brain is high and the water in the gray and white matter is similar, which makes it difficult for MRI to distinguish between gray and white matter, and therefore, the resolution of early PVL lesions by conventional MRI is also poor [11]. Amplitude-integrated electroencephalography (aEEG) is a novel CFM technique. Conventional EEG uses the international electrode placement method, which acquires multichannel signals, whereas aEEG acquires signals from a single electrode, commonly P3–P4 or C3–C4 electrodes, which are filtered through frequencies <2 Hz and >20 Hz and amplified in the rest of the range, while the amplitude is compressed to 0.1 V with an integrated velocity, as shown in Figure 1. Although aEEG is a compressed and simplified version of conventional EEG, studies have shown that aEEG electrical activity is more valuable for neurological assessment than conventional EEG. The aEEG waveform is a superimposed spectral band with a wide and narrow range of waveforms that are easy to grasp and to identify with precise standards [12, 13]. aEEG single-channel recordings not only reduce the cumbersome operations associated with conventional multilead EEG monitoring but also allow for a more accurate diagnosis of EEG activity. The aEEG single-channel electrodes are placed bilaterally in the parietal bone, which corresponds to the area supplied by the middle and posterior cerebral arteries, and is therefore sensitive to ischemia [14]. The aEEG instrument is also small and easy to use, allowing for continuous bedside monitoring without moving the critically ill preterm infant, making aEEG particularly suitable for use in the NICU [15].

At present, digital signal recording EEG technology has become the mainstream of EEG recording technology. Video EEG is a digital EEG technology based on dynamic EEG monitoring, which uses a video camera to simultaneously record images of the patient's daily activities and play back the EEG so that the doctor can simultaneously observe the child's clinical symptoms while observing the brain waves. Therefore, video EEG technology effectively avoids the short time, low positive rate, high cost, and storage difficulties of conventional EEG. EEG can objectively, directly, and rapidly reflect the state of brain function development and the degree of damage and determine the condition of the disease because there are different criteria for EEG for different gestational ages and different states. However, there are few studies on the early diagnostic value of EEG for periventricular white matter softening in preterm infants in the domestic literature. Therefore, this study aims to evaluate the value of VEEG as an early diagnostic indicator in screening preterm infants with PVL by monitoring VEEG of all preterm infants with suspected PVL and performing DWI of all preterm infants with suspected PVL (the gold standard) to confirm the diagnosis and to evaluate the value of VEEG as an early diagnostic indicator in screening preterm infants with PVL by comparing VEEG results with the gold standard through the evaluation method of clinical diagnostic test.

## 2. Data and Methods

### 2.1. Research Subjects

55 cases of premature infants with suspected PVL of 28–34 weeks' gestation, birth weight <2000 g, and hypoxia due to various reasons, who were transferred to the neonatal intensive care unit (NICU) of a medical university from January 2018 to January 2020, were selected. Actually, in this age range, the disease is most representative. The DWI monitoring results were used as the gold standard, and the diagnostic criteria were high signal in the periventricular white matter edema area and decreased ADC values. PVL group comprises 12 cases, 7 males and 5 females; the observation group comprises 43 cases, 26 males and 17 females, as shown in Table 1. Cranial ultrasound was performed to exclude cerebral ventricles and diseases such as internal bleeding.

### 2.2. Research Methods

The VEEG and DWI tests were performed simultaneously in the first week after birth. VEEG examination: the 64-guide VEEG provided by the Danish Veedi company, operated by professional physicians, sampling rate 128/min, time constant 0.1∼0.3, comembrane inhibition ratio >100 db, amplitude 10 *μ*V/mm, and paper speed 3.0 cm/s, adopted the recommendations of the American Association of Neurophysiology. A total of 8 electrodes in the international 10–20 system of Fp1, Fp2, C3, C4, O1, O2, T3, and T4, with binaural A1 and A2 as reference electrodes were traced in unipolar leads for 0.5–1 h, including at least one complete cycle of wakefulness, active sleep, and quiet sleep. W waves are confined to the central region, occasionally in the sagittal pars sagittal region, with high amplitude (20–200 *μ*V) positive spikes synchronized on one or both sides, often preceded and followed by a low-amplitude negative wave, with or without background wave abnormalities. The results are interpreted by two neurologists. 1.5 TMR scanner and standard head coil provided by Philips, the Netherlands, are used for DWI examination. Gastric sedation with 10% chloral hydrate intranasally was given 20 min before the examination. In all cases, the MRI scan was performed in axial, coronal, and sagittal planes. Postprocessing was performed using a GE workstation (SUN, ADW4.2). The isotropic DWI raw images were automatically generated by the machine, and the ADC maps were obtained by using the software. The ADC values of the corresponding brain tissues in the anterior, middle, and posterior parts of the white matter were measured and averaged. The ADC values and imaging reports were produced by two or more senior physicians.

### 2.3. Statistical Processing

The sensitivity, specificity, positive likelihood ratio, negative likelihood ratio, positive predictive value, negative predictive value, and compliance rate of the EEG diagnosis of PVL in preterm infants were analyzed according to the four-compartment table of the diagnostic test, and the sensitivity, specificity, positive likelihood ratio, negative likelihood ratio, positive predictive value, and compliance rate of the EEG diagnosis of PVL in preterm infants were analyzed according to the four-compartment table of the diagnostic test by kappa analysis. Calculate the concordance between the 2 screening methods for the diagnosis of PVL in preterm infants.

## 3. Comparison of Periventricular White Matter Softening in Preterm Infants

### 3.1. Periventricular White Matter Softening Factors

The occurrence of periventricular white matter softening is related to vascular anatomic factors (Figure 2). The periventricular area of the premature infant is the final blood supply area for the anterior, middle, and posterior cerebral arteries, where the metabolic rate and glucose demand are high. Due to immature vascular development, the periventricular area is the area with the least distribution of cerebral blood flow, and these areas are the most vulnerable to ischemic injury once systemic blood pressure drops, resulting in PVL [16]. After 32 weeks, the number of short-branched arteries gradually increases, the convergence of long- and short-branched arteries gradually increases, and the periventricular arterial terminal blood supply area gradually decreases, resulting in the frequency of PVL. The likelihood of PVL decreases with gestational age. The younger the gestational age is, the less mature the periventricular vasculature is, and the more likely the PVL is to occur [17]. Under normal circumstances, the cerebral vasculature in mature infants and adults has an autoregulatory function that constricts or dilates as cerebral perfusion pressure increases or decreases to maintain normal blood supply to the brain tissue [18].

However, premature infants, especially those with clinical instability (e.g., hypoxemia, hypocapnia, and severe disease requiring extracorporeal membrane pulmonary support), have immature autoregulation of cerebral blood flow, which results in passive pressure cerebral circulation; i.e., when systemic blood pressure decreases, cerebral blood flow also decreases and cerebral ischemia is likely to occur. This may be related to the following factors: (1) the immature development of the myenteric layer of the fetal cerebral artery in late pregnancy; (2) the narrow range of permissible fluctuations of blood pressure; and (3) the immature development of the blood-brain barrier, which disrupts the regulation of cerebral blood flow and results in passive pressure cerebral circulation. The white matter of preterm infants has three types of oligodendrocytes (OL): OL precursors, immature OL, and mature OL, and the latter mainly constituting the myelin sheath of the white matter of the brain [19]. During the onset of PVL in preterm infants (23–32 weeks), most of the lateral ventricular triangles in the white matter region of the preterm brain are highly active OL precursors. The normal development of OL precursor cells is also regulated by trophic factors and hormones secreted by astrocytes and functional development of astrocytes in preterm infants, which synthesizes and releases low amounts of b-FGF and IG protective nutrients and also promotes white matter vulnerability [20]. (3) Thyroid hormones are essential for normal brain development, and clinical data show that preterm infants have significantly lower levels of thyroid hormones and corticosteroids than full-term infants, which helps to explain the increased incidence of white matter damage in preterm infants [21].

The clinical picture of periventricular white matter softening in preterm infants is usually asymptomatic, lacking specific neurological signs and symptoms, and may present only as nonspecific symptoms such as poor response, muffled crying, decreased voluntary activity, intolerance to gastrointestinal feeding, and slow growth. The main clinical emphasis is on diagnosis, and the significance of early diagnosis, early symptomatic treatment, and early intervention is significant. Because clinical diagnosis is difficult and easily missed and misdiagnosed, it is important to know the brain function status of preterm infants at an early stage [22]. Therefore, craniocerebral imaging plays an important role in the early diagnosis of brain injury in preterm infants. Therefore, this diagnostic study was designed to verify whether the selected target test method, video electroencephalography (VEEG), can be used for early diagnosis of periventricular white matter softening in preterm infants and to preliminarily evaluate the usefulness of VEEG for early diagnosis of periventricular white matter softening in preterm infants [23]. All subjects were selected according to strict inclusion and exclusion criteria, video EEG and diffusion-weighted magnetic resonance examination were performed simultaneously and blindly, and the results are discussed below.

### 3.2. Imaging Diagnosis of PVL

The significance of imaging for the diagnosis of paraventricular white matter injury in preterm infants lies in the early detection of white matter injury, prompting the clinical clinic to avoid predisposing factors and treat them appropriately, and in the definitive diagnosis of the outcome of white matter injury, providing a basis for estimating prognosis and targeted interventions after the neonatal period [24]. Ultrasound, CT, and MRI are the main clinical methods used today. Ultrasound was first used by Hill in 1982 to diagnose PVL, and brain ultrasound (US) is still a good diagnostic tool, as the sensitivity of brain ultrasound differs depending on the pathologic classification. The pathological classification of periventricular white matter softening is mainly of two types: focal (c-PVL) and diffuse, with local PVL being characterized by acute necrosis of white matter oligodendrocyte precursors and the formation of multiple small vesicles at a later stage. Diffuse PVL, also known as diffuse white matter injury, is characterized by the apoptotic death of white matter oligodendrocyte precursors and, rarely, cystic lumen changes.

Focal periventricular white matter softening occurs predominantly in the peripheral zone of long-transverse arteries and is located deep in the white matter of the brain. It is characterized by focal necrosis of all cellular components and the formation of a vesicular cavity, most commonly located in the white matter adjacent to the lateral ventricular triangle and around the interventricular foramen. This site is the marginal zone between the middle and posterior cerebral arteries (white matter around the triangle) or between the long through-branch endings of the middle and anterior cerebral arteries (frontal white matter), respectively. The neuropathological evolution of focal periventricular white matter softening occurs 6 to 12 h after acute hypoxia-ischemia, as shown in Figure 3. Rapidly differentiating immature oligodendrocytes, especially around focal necrosis, were evident. After about 24–48 h, microglial infiltration appears at the necrotic site, accompanied by proliferation of mast astrocytes and endothelial cells. Foamy macrophages appeared around 5 d and became more obvious after 2 weeks; then 1–3 weeks later, the tissue dissolved and formed a small cystic cavity, often multifocal, which could be detected by cranial ultrasound when the diameter of the cavity was >0.5 cm. With further glial hyperplasia, the cystic cavity gradually shrinks and is no longer detected by ultrasound. Finally, focal myelin dysformation decreased white matter volume, and ventricular dilatation occurs, usually in the triangle of the lateral ventricles. Diffuse PVL is the predominant type of injury. Diffuse periventricular white matter softening is a milder form of white matter injury that is particularly likely to occur in very small preterm infants who have survived for a long time after birth. The neuropathologic evolution of diffuse periventricular white matter softening differs from that of focal periventricular white matter softening in that the cytologic hallmarks of diffuse periventricular white matter softening are nuclear condensation of oligodendrocytes and astrocytic hypertrophy, and the injury, although extensive, is not severe and does not affect all cellular components.

The main neuropathological features of this diffuse lesion, which is less prone to cystic cavity-like changes, are the diffuse loss of immature oligodendrocytes in the early stages of differentiation and the proliferation of mast astrocytes, with the consequence of reduced white matter volume and enlarged ventricles. Diffuse periventricular white matter softening is therefore primarily a specific injury of the oligodendrocyte precursor cells and cannot be detected by cranial ultrasound. The severity of local PVL lesions in ultrasound is generally classified into four grades according to the deVries classification: grade I: periventricular local echogenic enhancement (PVE) persists or is greater than 7 days, after which no cystic lesions appear; grade II: periventricular local echogenic enhancement, which then turns into local small cystic lesions; grade III: extensive periventricular echogenic enhancement, which then turns into extensive cystic lesions; and grade IV: extensive cystic lesions, which then turns into small cystic lesions. Grade V: widespread periventricular echogenic enhancement involving subcortical white matter, which later turns into periventricular and subcortical diffuse cystic cavity injury. According to the grading of lesions, PVL cystic cavity formation is late, usually in 2–4 weeks after birth, which is consistent with pathological changes. c-PVL is less common clinically than diffuse PVL, accounting for about 30% of PVL, and mostly appearing in 2–4 weeks after birth. The specificity of cranial CT for the early diagnosis of PVL is poor. For the diagnosis of PVL by CT, it was concluded that PVL could not be diagnosed by periventricular hypodensity alone in 17 cases of preterm infants at 40 weeks of corrected gestational age because 40% of normal newborns could have similar behavior. This is because the white matter of preterm infants is not yet myelinated and shows a generalized low density, and when the periventricular white matter is damaged by hypoxia, it is difficult to identify it by CT. The sensitivity and specificity for the early diagnosis of white matter lesions are low, and the diagnostic significance is limited.

Magnetic resonance imaging (MRI), as a noninvasive technique, has good density resolution of the gray and white matter of the brain and can be used to examine the multiaxial plane, including cross-sectional, coronal, and sagittal plane, which is convenient for lesion characterization, localization, and quantification, without the harm of X-ray radiation. In the early stage of PVL, periventricular white matter damage can be manifested as T1W1 low signal and T2W1 high signal in the lesion area, but because the white matter myelin is not formed in preterm infants, this brain white matter is high in water content, also manifested as T1W1 low signal and T2W1 high signal, as shown in Figure 4. It is not as good as B-ultrasound and DWI, so the diagnostic value of routine MRI scan in early PVL is not great, and MRI is more valuable in the diagnosis of late PVL, which can show decreased white matter volume, enlarged ventricles, ventricular wall irregularities, neuronal cell glial hyperplasia, and delayed myelin formation. Therefore, routine MRI is usually used to evaluate development in late neonatal or infant follow-up.

### 3.3. Video EEG Diagnosis

In summary, the commonly used imaging methods such as brain ultrasound, cranial CT, and routine MRI cannot diagnose PVL at an early stage, and the clinic needs to look for other examination methods to achieve early diagnosis. The diffusion-weighted imaging (DWI) technique developed in recent years has changed this situation. Dispersion-weighted MRI is an imaging technique that reflects the irregular movement of water molecules in tissues and is currently the only noninvasive method capable of detecting the diffusion movement of water molecules in human tissues, which can reflect the internal characteristics of the microstructure of tissues and provide unique information about the functional state of the brain at the level of water molecules. The ADC value of the molecule is used to make an early diagnosis of the disease.

It has been found that, by using diffusion-weighted imaging techniques of MRI, the paraventricular diffusion coefficient can be reduced in the early stage of PVL, which is cytotoxic brain edema with limited water molecule diffusion. In contrast, conventional MRI shows abnormal T2W1 signal only after the appearance of c-PVL. It has been shown that DWI can detect acute lesions at an early stage and can reflect the white matter lesions in the brain by using the apparent dispersion coefficient (ADC), which increases the ADC and decreases the diffusion of water molecules and the signal of diffusion-weighted images, while the diffusion of water molecules slows down and the ADC decreases and the signal of DWI increases, indicating the occurrence of cytotoxic edema. The results also demonstrate that DWI can be used for early diagnosis of periventricular white matter softening in preterm infants. The results of this study also prove that DWI can diagnose periventricular white matter softening at an early stage. The data of this group are as follows. It shows a group of 12 PVL cases with high signal on diffusion-weighted images (see Figure 5) and reduced ADC values. Although DWI can diagnose PVL at an early stage, DWI equipment and examination are expensive, long lasting, and noisy, and children need to be transported to the MRI room, which is not conducive to the examination of critically ill children. Premature infants who are critically ill or who do not have the financial means to undergo DWI can be diagnosed early, which is of great clinical importance for early treatment.

Video electroencephalography (VEEG), a more advanced electroencephalography technique, has been widely used at home and abroad in the past decade for the qualitative and typological diagnosis of epilepsy and has been gradually applied to neonatal brain injury in recent years due to its superiority. It has been found that video EEG technology can easily record the clinical manifestations of neonatal seizures and their EEG changes, which is beneficial to the correct diagnosis and treatment of this disease. It is believed that video EEG can dynamically reflect the state of brain function in a timely manner and has a high correlation with US and MRI in determining the time of cerebral hypoxia-ischemia in preterm infants, which can compensate for the deficiencies of the two and achieve the purpose of early detection and diagnosis, thus greatly reducing the disability rate of preterm infants. From an EEG point of view, the newborn is a very special period. From prematurity to full term, the developmental pattern of EEG background activity roughly evolves from discontinuous patterns to alternating patterns and finally to continuous patterns. In normal neonates, there can be a variable number of spikes and spikes in the EEG. The more immature the brain is, the greater the number of spikes and spikes, and the more the they appear in the frontal, central, or temporal regions.

Because the physiologic parameters of the wake-sleep state are often inconsistent in neonates, especially in preterm infants, there is a great deal of reliance on the observation of clinical behavior to determine the state. The EEG technician should be at the bedside at all times to observe and mark in real-time events such as postural changes, limb movements, facial movements, eye openings, and suspicious seizures. The advantages of VEEG over ordinary EEG are as follows: (1) it helps the physician to identify artifacts more accurately because EEG is a very weak signal that can be easily disturbed by external factors such as the patient's slightest movement or the movement of others; (2) more direct observation of the patient. These two points are the main differences between video EEG and ordinary EEG, which provide more comprehensive and accurate information. VEEG has a complete case management function, which can store, query, and statistically analyze thousands of cases, and the results can be stored on CD-ROM or USB removable hard disk for easy academic communication.

## 4. Results and Discussion

All preterm infants enrolled in the study underwent brain ultrasound before DWI and VEEG because although brain ultrasound has its limitations in the early diagnosis of PVL, it is the diagnostic method of choice in the diagnosis of IVH, and the important reason is that brain ultrasound has specific diagnostic value for lesions in the central part of the brain. In preterm infants, especially those under 32 weeks of gestational age, there is a germinal matrix (GM) under the periventricular ventricular membrane. The vascular wall of the GM is composed of an irregular layer of endothelial cells, which lacks collagen and elastic fiber support, and there is no direct support structure between the periventricular tissues and the wall of the GM.

The small veins in the GM layer are U-shaped, and this orientation slows down the blood flow and makes it easy to infarct, increase capillary pressure after small vein embolism, and cause blood vessel rupture and bleeding. Therefore, the vessels in the GM layer are susceptible to damage from hypoxia, fluctuating blood pressure, and other factors. When there is too much blood in the ventricle, the ventricle widens and further develops, damaging the tissues around the ventricle, and the enlargement of the ventricle causes damage to the paraventricular white matter, which is about 26% of PVL combined with intraventricular hemorrhage. Therefore, brain ultrasound screening is required to exclude preterm infants with intraventricular hemorrhage in order to ensure the authenticity of the test results.

Studies have shown that most acute EEG abnormalities are transient and resolve quickly, so the timing of EEG monitoring in preterm infants is important, with the most predictive EEG occurring in the first week of life. Video EEG during PVL is commonly characterized by changes in the EEG background and the presence of epileptiform discharges, with specific EEG changes in the form of PRSW, most commonly observed on postnatal days 5 to 8.3. The abnormalities will gradually disappear after ∼4 weeks. Therefore, this diagnostic test should be performed within one week after birth to detect abnormalities in the video EEG in time, so as not to miss the test, which may result in missed or misdiagnosis. In this experiment, VEEG was used to monitor all cases in the three groups, as shown in Figure 6, and it was synchronized with DWI, but because DWI examination requires sedation, which may affect the EEG results, VEEG examination was given priority over DWI. Positive cases of VEEG mainly showed suppressed background activity: prolonged interburst interval in 4 male cases, abnormal spikes in 2 female cases, and turbulent waves that did not correspond to the gestational age. Normal spikes and spike waves can be seen in newborns of all stages and decrease with EEG maturation.

In this diagnostic test, VEEG monitoring indicated PRSW waves (see Figure 7). To ensure the accuracy of the diagnosis, VEEG monitoring was repeatedly performed with different speeds, amplitudes, and frequencies of paper travel. The lack of PRSW in early preterm EEG was reported to be associated with favorable motor development in preterm infants (98.2%) and demonstrated the value of PRSW in the early diagnosis of PVL with a sensitivity of 98% and a specificity of 84%. PRSW waves were seen in 13 positive cases screened by VEEG, of which 10 cases were diagnosed with PVL by DWI. Because abnormal background activity is a sign of cortical injury and periventricular white matter softening often affects the white matter, PRSW waves and abnormal background activity are often seen together. In the negative group, there were also signs of background activity suppression, including reduced wave amplitude that did not correspond to the corresponding week of gestation or the presence of frontal spikes.

The results of the four-compartment diagnostic test were calculated (see Figure 8): the sensitivity of video EEG for PVL diagnosis was 83%, the specificity 93%, the missed rate 17%, and the misdiagnosis rate 7%. Sensitivity and specificity are the main indicators of the effectiveness of diagnostic tests and are used to explain how consistent the results obtained by diagnostic tests are with actual conditions. Sensitivity refers to the ability of diagnostic tests to correctly diagnose people with actual illness as a patient. The difference sensitivity between the male and female can also be seen. The results of this test indicate that the sensitivity was 83%, which is slightly lower than the literature. In addition, since the hospital is temporarily unable to perform bedside electroencephalography (EEG), children were selected to be in stable condition, without frequent apnea or premature infants not on ventilator treatment. The specificity refers to the ability of a diagnostic test to correctly diagnose people who are not actually sick as nonpatients, and the results of this test can be considered to have a high specificity and a low rate of misdiagnosis. As a result, Oliver collected 605 cases of preterm infants within a week of birth over a period of 4 years. It has been reported in the literature that PVL is the main factor for cerebral palsy in surviving preterm infants, and it has been suggested that the occurrence of PRSW waves is related to cerebral palsy, so Oliver collected EEG data of 605 cases of preterm infants within one week after birth over a period of 4 years to verify the sensitivity and specificity of PRSW waves for PVL diagnosis. The cases were divided into two groups: group I <27 W and group II: 28∼31 W. Statistical analysis of EEG results showed that PRSW wave was a high specificity indicator for both groups: 100% for group I and 99.8% for group II; the sensitivity of PRSW wave for PVL diagnosis depended on gestational age: 32.4% for group I and 87.8% for group II. It is concluded that PRSWW is an early and highly specific indicator of PVL in preterm infants.

The test has a misdiagnosis rate of 7% and a missed diagnosis rate of 13%. The reason for the misdiagnosis is that VEEG reflects the functional state of the brain, so whenever a preterm infant has a history of hypoxic-ischemic disease, there is a possibility that the corresponding brain wave changes may occur at an early stage. To date, the mechanism of PRSW wave generation is not clear. Therefore, PRSW can also be detected in normal preterm infants, suggesting that neonatal video EEG should be followed dynamically in clinical practice when conditions permit, in order to avoid clinical misdiagnosis.

## 5. Conclusion

Periventricular white matter softening in preterm infants can lead to severe sequelae and greatly affect the quality of life of preterm infants, and early diagnosis has high clinical significance and value. The purpose of this study is to select the diagnostic test scientifically and rationally, to interpret and evaluate the results of the diagnostic test correctly, and to evaluate the selected diagnostic method. Although DWI is a sensitive method for early diagnosis of PVL, it is not suitable for critical preterm infants. Therefore, according to clinical research data and the basic hardware conditions of our hospital, video EEG was chosen as the target diagnostic test method to explore whether VEEG can be used for early diagnosis of PVL. The results of this diagnostic test suggest that the sensitivity and specificity are high, and combined with the advantages of video EEG examiner, noninvasiveness, safety, feasibility, and cheapness, this test believes that video EEG can be used as an auxiliary test for early diagnosis of PVL. After EEG, for some critically ill preterm infants who are not suitable or financially unable to undergo DWI, it may be possible to use the EEG as an indicator for preliminary screening, in order to make a preliminary diagnosis of periventricular white matter softening in preterm infants and to suggest necessary and timely clinical interventions.

## Figures and Tables

**Figure 1:** Symptoms of periventricular white matter softening in preterm infants.

**Figure 2:** Flow of factor analysis of periventricular white matter softening.

**Figure 3:** Changes in cerebral oxygen consumption.

**Figure 4:** Signal variation in T1W1 and T2W1.

**Figure 5:** Diffusion-weighted signal variation.

**Figure 6:** EEG results under video detection.

**Figure 7:** VEEG monitoring to cue PRSW waves.

**Figure 8:** Calculation results of the four-compartment table for diagnostic tests.

**Table 1:** The general information of selected patients.

Group	Average age (weeks)	Gender (male/female)	Disease duration (month)	Injury part	
				Left	Right
Control	28–34	7/5	0.83 ± 0.12	18	22
Observation	28–34	26/17	0.76 ± 0.07	18	22

## Data Availability

The data used to support the findings of this study are available from the corresponding author upon request.
